This article has been retracted.

# miR-1301 inhibits hepatocellular carcinoma cell migration, invasion, and angiogenesis by decreasing Wnt/*β*-catenin signaling through targeting BCL9

**DOI:** 10.1038/cddis.2017.356

**Published:** 2017-08-17

**Authors:** Chao Yang, Yonghua Xu, Feng Cheng, Yuanchang Hu, Shikun Yang, Jianhua Rao, Xuehao Wang

**Affiliations:** 1 Department of Liver Surgery/Liver Transplantation Center, The First Affiliated Hospital of Nanjing Medical University; Key Laboratory on Living Donor Liver Transplantation of National Health and Family Planning Commission of China, Nanjing, China; 2 Department of General Surgery, Yancheng City No.1 People’s Hospital/The Fourth Affiliated Hospital of Nantong University, Yancheng, China

## Abstract

Metastasis is the major cause of the poor prognosis of hepatocellular carcinoma (HCC), and increasing evidence supports the contribution of miRNAs to cancer progression. However, the exact relationship between the level of miR-1301 expression and HCC cell migration, invasion, and angiogenesis remains largely unknown. Quantitative PCR was used to evaluate the level of miR-1301 expression in HCC tissues and cell lines. Transwell and tube-formation assays were used to measure the effects of miR-1301 on HCC cell migration and invasion, and angiogenesis, respectively. Luciferase reporter assays and western blotting were used to confirm the miR-1301 target genes. We found that miR-1301 was significantly downregulated in HCC tissues and cell lines. Low miR-1301 expression was associated with tumor vascular invasion and Edmondson grade. Gain- and loss-of-function assays demonstrated that miR-1301 inhibited the migration, invasion, epithelial–mesenchymal transition, and angiogenesis of HCC cells *in vitro* and *in vivo*. BCL9, upregulated in HCC tissues compared with matched adjacent normal tissues, was inversely correlated to miR-1301 levels in HCC tissues. Through reporter gene and western blot assays, BCL9 was shown to be a direct miR-1301 target. BCL9 overexpression could partially reverse the effects of miR-1301 on HCC cell migration and invasion. Most importantly, miR-1301 overexpression markedly suppressed the death of xenograft mouse models of cancer by reducing tumor load, metastasis, and host angiogenesis by downregulating BCL9, *β*-catenin, and vascular endothelial growth factor expression in tumor cells. Our observations suggested that miR-1301 inhibits HCC migration, invasion, and angiogenesis via decreasing Wnt/*β*-catenin signaling through targeting BCL9, and might be a therapeutic target for HCC.

Hepatocellular carcinoma (HCC) is the fifth most frequent malignancy and the second leading cause of cancer-related mortality worldwide. The incidence of HCC is particularly high in Asia, where the high prevalence of hepatitis B and C strongly predisposes individuals to developing chronic liver disease, and subsequently HCC.^1, 2^ There are no obvious symptoms during the early stages of the disease; HCC patients are commonly diagnosed at advanced or unresectable stages.^3, 4^ Metastasis after curative resection is the most challenging burden for HCC treatment;^5^ however, the underlying mechanisms of HCC metastasis are largely unknown.

MicroRNAs (miRNAs) are a class of evolutionarily conserved small noncoding RNAs that usually suppress the expression of protein-coding genes by targeting their 3′-untranslated region (3′-UTR).^6^ As post-transcriptional regulators of gene expression, miRNAs are involved in regulating many central biological processes, such as cell proliferation, differentiation, apoptosis, cell cycle progression, migration, and tumorigenesis.^7, 8, 9^

Accumulating evidence has suggested that miR-1301 might play critical roles in human cancers. For example, Fang *et al.*^10^ found that miR-1301 was downregulated in HepG2 cells, and that its overexpression inhibited cell migration and invasion, and induced apoptosis, suggesting miR-1301 is a tumor suppressor. Conversely, Liang *et al.* found that miR-1301 was upregulated in liver cancer cells and tissues, where it promoted cell proliferation, migration, and angiogenesis. Mechanistic analysis has shown that miR-1301 inhibits the tumor suppressor KLF6-FL, promoting tumor progression.^11^ Bi *et al.*^12^ indicated that forced miR-1301 expression promoted prostate cancer proliferation by inhibiting PPP2R2C. However, the exact roles of miR-1301 in HCC progression and metastasis remain unclear as do the molecular mechanisms in which it is involved.

The canonical Wnt/*β*-catenin pathway has been implicated in the pathogenesis of a broad range of human cancers,^13^ and its components have emerged as targets for cancer therapy.^14^ Numerous coactivators of *β*-catenin transcription have been identified, including B-cell lymphoma 9 (BCL9), its homolog BCL9-like, Pygopus and others.^15, 16^ The human *BCL9* gene was originally identified in lymphoblastic leukemia cells harboring a chromosomal translocation that led to its transcriptional activation.^17^ BCL9 is overexpressed in a variety of malignancies, and as a component of the aberrantly activated Wnt signaling pathway, promotes cell proliferation, migration, invasion, and metastasis of tumor cells.^18, 19^ A previous study identified that BCL9-2 promotes the early stages of intestinal tumor progression.^20^ However, a functional link between miR-1301 and the Wnt pathway coactivator BCL9 in association with HCC migration, invasion, and angiogenesis has not been established.

In this study, we report an inhibitory role of miR-1301 in HCC progression. We show that both *in vivo* and *in vitro* miR-1301 suppresses tumor migration invasion and angiogenesis by targeting multiple angiogenesis-inducing genes, including BCL9, *β*-catenin, and vascular endothelial growth factor-A (VEGF-A), thus highlighting a dual role for miR-1301 in tumor metastasis.

## Results

### miR-1301 is downregulated in HCC tissues and cell lines

To determine whether miR-1301 was abnormally regulated in HCC tissues, miR-1301 expression was examined in 60 pairs of HCC and adjacent normal tissues by quantitative PCR (qPCR). As shown in Figure 1a, miR-1301 expression was significantly lower in human HCC samples than in adjacent normal tissues. We then investigated the association between the miR-1301 expression and the clinicopathological features of HCC. All HCC patients involved in this study were divided into a high miR-1301 expression group and a low miR-1301 expression group, using the mean value of miR-1301 expression as the cutoff point. As indicated in Table 1, 39 cases (65%) were in the low miR-1301 group, while 21 cases (35%) were in the high miR-1301 group. Decreased miR-1301 expression was significantly associated with tumor vascular invasion and Edmondson grade (Table 1). However, no statistically significant association between miR-1301 expression was found with age, gender, tumor size, alpha-fetoprotein, HBV infection, or cirrhosis (Table 1). Further experiments showed that several HCC cell lines, including Hep3B, HepG2, SMMC-7721, and Huh-7 also had low miR-1301 levels. By contrast, the normal liver cell line LO2 had high miR-1301 levels (Figure 1b). Next, we chose three paired HCC and noncancerous tissues for fluorescence *in situ* hybridization (FISH) analysis, and found consistent results (Figure 1c). The significant downregulation of miR-1301 in HCC tissues and cell lines supports its role as a tumor suppressor in HCC.

These results indicated that miR-1301 was downregulated in both HCC tissues and cancer cell lines. To investigate the impact of miR-1301 on tumor migration, invasion and angiogenesis, we constructed both miR-1301 overexpression and knockdown HCC cell lines (Figures 1d and e). As shown, miR-1301 expression was decreased by approximately 95% in targeted SMMC-7721 cells, and increased approximately 20-fold in Huh-7 cells.

### miR-1301 regulates tumor angiogenesis *in vitro*

To confirm that miR-1301 is a potential angiogenesis suppressor in HCC, we investigated the influence of miR-1301 on human umbilical vein endothelial cell (HUVEC) tube formation, migration, and invasion *in vitro*.

Tube-formation assays with HUVECs were performed in different conditioned media (miR-1301 inhibitor, pre-miR-1301, or empty vector). Compared with control cells, silencing miR-1301 increased the tube-forming capacity of HUVECs, whereas miR-1301 overexpression dramatically reduced tube-forming capacity (Figures 2a and d).

Next, we used cell migration and Matrigel invasion assays to investigate the effects of miR-1301 on HUVEC migration and invasion. Our data revealed that HUVECs migration was enhanced by miR-1301 knockdown in SMMC-7721 and Huh-7 cells, whereas migration was suppressed by miR-1301 overexpression in SMMC-7721 and Huh-7 cells (Figures 2b and e). Additionally, compared with control cells, silencing miR-1301 dramatically boosted HUVECs invasiveness, whereas miR-1301 upregulation inhibited HUVECs invasiveness (Figures 2c and f).

### miR-1301 negatively regulates HCC cell migration, invasion, and EMT

To confirm that miR-1301 functions as a tumor suppressor in HCC, we investigated the influence of miR-1301 on the migration and invasion of HCC cells *in vitro*. We used cell migration and Matrigel invasion assays to investigate the effects of miR-1301 on HCC cell migration and invasion. Our data indicated that cell migration was enhanced when miR-1301 was downregulated, whereas migration was suppressed by miR-1301 overexpression in Huh-7 and SMMC-7721 cells (Figures 3a and c). Additionally, compared with the control cells, miR-1301 silencing in Huh-7 and SMMC-7721 cells dramatically boosted cell invasion, whereas miR-1301 upregulation inhibited Huh-7 and SMMC-7721 cell invasion (Figures 3b and d). Wound healing assays also supported the conclusion that miR-1301 suppressed the migration of HCC cells. Additionally, the miR-1301-inhibitor significantly accelerated the migration of HCC cells, while cells cultured in pre-miR-1301 medium were distinctively less migratory (Figure 3e). We further examined the protein levels of epithelial–mesenchymal transition (EMT)-related factors. Western blot data indicated that after miR-1301 upregulation in SMMC-7721 and Huh-7 cells, E-cadherin levels were increased, while Vimentin and Slug levels were reduced. Silencing miR-1301 expression showed the opposite results (Figure 3f). These data suggest miR-1301 suppresses cell migration, invasion, and EMT in HCC cells.

### VEGF-A expression is inhibited by miR-1301

SMMC-7721-NC, SMMC-7721-miR-1301-inhibitor, SMMC-7721-pre-miR-1301, Huh-7-NC, Huh-7-miR-1301-inhibitor, and Huh-7-pre-miR-1301 cells were used to test the levels of VEGF-A, which is the most important angiogenic factor influencing the vasculature and angiogenesis. As shown in Figure 4a, compared with SMMC-7721-NC cells, VEGF-A mRNA levels in the SMMC-7721-miR-1301-inhibitor cells were increased by approximately 90%. Compared with the Huh-7-NC cells, VEGF-A mRNA levels in the Huh-7-pre-miR-1301 cells were decreased by approximately 40%. Similarly, the protein levels of VEGF-A were increased in SMMC-7721-miR-1301-inhibitor and Huh-7-miR-1301-inhibitor cells compared with SMMC-7721-NC and Huh-7-NC cells, and were further decreased in SMMC-7721-pre-miR-1301 and Huh-7-pre-miR-1301 cells compared with SMMC-7721-NC and Huh-7-NC cells (Figure 4b). We also used ELISA to detect secreted VEGF-A protein in the supernatants of the above cell lines. As expected, miR-1301 knockdown increased secreted VEGF-A levels, while miR-1301 overexpression decreased secreted VEGF-A levels (Figure 4c).

### BCL9 is upregulated in human HCC tissues and cell lines

To examine the association between miR-1301 and BCL9, we further analyzed BCL9 expression in the 60-paired human HCC and adjacent normal tissues by qPCR. As shown in Figure 5a, BCL9 was upregulated in HCC tissues. qPCR was also used to determine the level of BCL9 expression in both the HCC cell lines and LO2 cells; these results demonstrated that BCL9 was more highly expressed in HCC cell lines than LO2 cells (Figure 5b). We next examined BCL9 expression in six paired HCC and healthy tissues by immunohistochemistry. As shown in Figure 5c, this assay also showed increased BCL9 expression in HCC tissues compared with adjacent normal tissues.

### The BCL9 3′-UTR is a target of miR-1301

TargetScan, PicTar, and miRanda were used to analyze potential miR-1301 targets. Candidates recovered from these algorithms were analyzed by Cancer Gene Index (https://wiki.nci.nih.gov/display/cageneindex/Cancer+Gene+Index+End+User+Documentation) to search for metastasis and angiogenesis promoters. Among them, we were particularly interested in BCL9, because it promotes tumor progression by conferring enhanced metastatic and angiogenic properties to cancer cells.^18^ As indicated in Figure 5d, BCL9 was a putative target of miR-1301, and perfect base pairing was observed between the seed sequence of mature miR-1301 and the BCL9 3′-UTR. To demonstrate the computational prediction results, qPCR and western blotting were used to determine BCL9 expression subsequent to changes in miR-1301 expression. As shown in Figures 5e and f, we found that miR-1301 overexpression was associated with decreased BCL9 mRNA and protein expression, whereas silencing miR-1301 showed the opposite results. A luciferase reporter assay was then used to validate whether BCL9 was a direct target of miR-1301. Wild-type (WT) and mutant (MUT) versions of the BCL9 3′-UTR – the latter containing site-directed mutations in the putative miR-1301 target sites – were cloned into reporter plasmids. Ectopic miR-1301 expression markedly suppressed luciferase activity from the WT reporter but not from the MUT reporter, suggesting that the 3′-UTR of BCL9 is targeted by miR-1301 and that the point mutations in this sequence abolished this interaction (Figure 5g).

### BCL9 is inversely correlated with miR-1301 in HCC

As we found that BCL9 was a direct miR-1301 target gene that was involved in the miR-1301-mediated malignant phenotypes of HCC cells *in vitro*, we speculated that miR-1301 downregulation might contribute to BCL9 upregulation in HCC tissues. To verify this speculation, we conducted qPCR to examine BCL9 expression in HCC tissues and adjacent normal tissues, and analyzed the correlation between the miR-1301 and BCL9 levels in HCC tissues. qPCR data indicated that BCL9 was upregulated in HCC tissues compared with adjacent normal tissues (Figure 5a). Moreover, we found that the BCL9 levels were inversely correlated with miR-1301 levels in HCC tissues (Figure 5h). These findings suggested that BCL9 upregulation in HCC may be caused by miR-1301 downregulation.

### BCL9 overexpression partially reverses the effects of miR-1301 on HCC migration and invasion

To further illustrate that miR-1301 affects the migration and invasion of HCC cells by regulating BCL9, Huh-7 cells were transfected with pre-miR-1301 lentivirus for 72 h, followed by transfection with LV-BCL9. BCL9 overexpression was verified by western blotting (Figures 6a and c). SMMC-7721 cells were transfected with miR-1301 inhibitor lentivirus for 72 h, followed by transfection with BCL9-shRNA. BCL9 downregulation was also verified by western blotting (Figures 6b and d). Through cell migration and Matrigel invasion assays, we found that ectopic BCL9 expression reversed the suppression of migration and invasion caused by miR-1301 overexpression (Figure 6e). In SMMC-7721 cells, the similar rescue effects were also observed, in which phenotypes caused by miR-1301 silencing were mitigated by BCL9 downregulation (Figure 6f).

### miR-1301 regulates the Wnt/*β*-catenin pathway through BCL9

Previous studies have reported that the *β*-catenin/BCL9 complex is an important target for cancer therapy;^21^ hence, we further conducted western blotting experiments to examine *β*-catenin levels in SMMC-7721 and Huh-7 cells after miR-1301 overexpression and knockdown. We found that the level of *β*-catenin protein expression was significantly decreased in the pre-miR-1301 group compared with the miR-NC group, whereas miR-1301 knockdown showed the opposite results (Figure 5f). Taken together, these results suggested miR-1301 might regulate Wnt/*β*-catenin signaling through BCL9, which may have also resulted in the altered expression of angiogenesis-associated proteins.

### miR-1301 inhibits HCC migration, invasion, and angiogenesis *in vivo*

To investigate whether miR-1301 overexpression could suppress HCC metastasis *in vivo*, SMMC-7721 cells with miR-1301 knockdown, miR-1301 overexpression and negative control were injected into the tail vein of BALB/c nude mice. As shown in Figure 7a, after 6 weeks, bioluminescence imaging revealed that the nude mice that were injected with miR-1301 knockdown cells exhibited more distant metastases. While some distant metastases were observed in the negative control group, the incidence in the group injected with miR-1301-overexpressing SMMC-7721 cells was significantly lower. The same results were observed in Huh-7 cells (Figure 7b). Taken together, these results suggested that miR-1301 overexpression suppressed HCC metastasis *in vivo*, consistent with our *in vitro* results.

We then isolated several organs that were reported to have higher HCC metastatic tropism and detected BCL9, VEGF-A, and CD31 expression by immunohistochemistry. The results showed that the number of CD31-positive microvessels was dramatically increased (approximately 4-fold) by the SMMC-7721-miR-1301 inhibitor, whereas SMMC-7721-pre-miR-1301 decreased the number of CD31-positive microvessels by 70% compared with controls (Figure 7c). Similar trends were observed with respect to BCL9 and VEGF-A expression in tumors (Figures 7d and e). We also detected miR-1301 expression in the metastatic tumors derived from nude mice by qPCR. As shown in Figures 7f and g, miR-1301 expression was increased in the pre-miR-1301-treated group, while the opposite effect was shown in the miR-1301-inhibitor-treated group. Additionally, BCL9 expression was determined by western blotting. We found that the level of BCL9 expression was decreased in the pre-miR-1301-treated group, whereas BCL9 protein levels were increased in the miR-1301-inhibitor-treated group (Figure 7h).

## Discussion

Despite the overwhelming evidence that has highlighted the clinical significance and prognostic implication of aberrant BCL9 expression in multiple cancer types, the molecular mechanisms underlying BCL9 activity in HCC remain elusive. In this study, we propose a novel role for miR-1301 in coordinating the expression of BCL9 in HCC cells. First, we showed that oncogenic BCL9 is a *bona fide* miR-1301 target in HCC. We also observed reduced miR-1301 expression in HCC specimens and cell lines concomitantly BCL9 was upregulated in HCC tissues and cell lines. We then demonstrated that miR-1301 overexpression downregulates BCL9 mRNA and protein expression, which was correlated with decreased cell migration and angiogenesis. Hence, we conclude that one of the molecular mechanisms by which miR-1301 inhibits cell migration, invasion, and angiogenesis is through negative regulation of the oncogene BCL9.

A biological function for miR-1301 in tumorigenesis has recently been proposed but the underlying mechanism remains largely unknown. Very recently, a small number of reports have shown varied expression in different cancer types and clinical specimens. miR-1301 overexpression was observed in prostate cancer, squamous cell carcinomas, and colorectal cancer with liver metastasis.^12, 22, 23^ Liang *et al.*^11^ found that miR-1301 was highly expressed in liver cancer cell lines as well as clinical specimens, and that miR-1301 overexpression promoted cell migration and angiogenesis by targeting the tumor suppressor KLF6-FL. Conversely, another report showed that miR-1301 was downregulated in HepG2 cells, and that miR-1301 inhibited the migration and invasion of HepG2 cells; they also showed that apoptosis was triggered after transfecting miR-1301 mimics.^10^ In agreement with this finding, our results revealed that the miR-1301 levels were significantly reduced in HCC tissues compared with paired adjacent normal tissues. Moreover, miR-1301 inhibited the migration, invasion, EMT and angiogenesis of HCC cells *in vitro* and *in vivo*, suggesting that miR-1301 downregulation is involved in HCC progression, and that miR-1301 may be a prognostic indicator for HCC patients. Our study further confirmed that miR-1301 acts as a tumor suppressor in HCC.

Cancer cells of epithelial origin can metastasize by transforming into cells with a mesenchymal phenotype, which is called EMT.^24, 25^ During EMT, epithelial cells gradually lose their connection to the basement membrane, and with increased invasive potential, can degrade the extracellular matrix.^24, 25^ Moreover, EMT is also characterized by decreased expression of cell adhesion molecules such as E-cadherin, the transformation of Cytokeratin into Vimentin, and the change to a mesenchymal morphology.^24, 25^ Thus, EMT is important for cancer migration and invasion.^25^ In this study, miR-1301 overexpression significantly increased E-cadherin expression, while reducing the levels of Vimentin and Slug proteins, indicating that EMT was inhibited. These findings were consistent with our migration and invasion data.

Tumor angiogenesis is crucially dependent on communication between the tumor and the associated endothelium.^26^ The migration, invasion, and tube formation of HUVECs are important processes mirrored during tumor angiogenesis.^27^ Here, we describe a role for miR-1301 in inhibiting angiogenesis, which was supported by a number of *in vitro* and *in vivo* experiments. miR-1301 depletion in HCC cells promoted HUVEC migration, invasion, and tube formation *in vitro* and increased the micro-vessel density *in vivo*. By contrast, enhanced miR-1301 expression suppressed these effects. Further experiments revealed that miR-1301 could attenuate tumor angiogenesis by downregulating VEGF-A expression. These results strongly suggest that miR-1301 downregulation enhances HCC progression.

We further identified BCL9 as a novel miR-1301 target gene, finding that miR-1301 could inhibit BCL9 protein expression in HCC cells. Previous studies have revealed that dysregulated BCL9 expression is an oncogenic mechanism of Wnt pathway activation.^28^ BCL9 serves fundamental roles in tumor progression by increasing tumor load, metastasis, angiogenesis, and invasion through regulating Wnt target genes.^29, 30^ We examined BCL9 expression in HCC tissues, and found that the BCL9 levels were inversely correlated with miR-1301, supporting the hypothesis that miR-1301 downregulation may contribute to BCL9 upregulation in HCC. *In vivo* studies further showed that mice bearing pre-miR-1301 SMMC-7721 and Huh-7 cells had fewer gastrointestinal and liver metastases than miR-1301-NC mice. The metastatic ability of SMMC-7721 and Huh-7 cells significantly decreased when endogenous miR-1301 was upregulated, compared with SMMC-7721-NC and Huh-7-NC cells. miR-1301 overexpression significantly inhibited HCC cell metastasis in nude mice, and protected the mice from tumor induced death. These findings further suggest that miR-1301 inhibits HCC metastasis by inhibiting BCL9.

In summary, our data revealed that miR-1301 was downregulated in HCC and that miR-1301 overexpression inhibited HCC migration, invasion, EMT, and angiogenesis. Additionally, miR-1301 downregulated BCL9 expression through direct binding to the BCL9 3′-UTR. We also found that miR-1301 inhibited the migration, invasion, and angiogenesis of HCC cells by targeting BCL9, which decreased Wnt/*β*-catenin signaling. In general, our findings provide a new prospective on the molecular targets for HCC treatment; however, the exact mechanism of how miR-1301 inhibits HCC metastasis is still not fully understood, and will be addressed in future work.

## Materials and methods

### Ethics statement

This study was approved by the Ethics Committee of the Nanjing Medical University and written informed consent was obtained from all enrolled patients.

### Tissue samples and cell lines

A total of 60-paired HCC and adjacent normal tissues were obtained from patients who were treated with curative hepatectomy at The First Affiliated Hospital of Nanjing Medical University, China, and samples were immediately frozen in liquid nitrogen for RNA and protein extraction. The clinicopathological characteristics of the patients were independently diagnosed by two professional pathologists.

All human HCC cell lines Hep3B, HepG2, SMMC-7721, and Huh-7, and the human normal liver cell line (LO2) were purchased from the Chinese Academy of Sciences (Shanghai, China) and were cultured in Dulbecco’s modified Eagle’s medium (DMEM; Life Technologies, Carlsbad, CA, USA) supplemented with 10% fetal bovine serum (Life Technologies) and antibiotics (100 U/ml penicillin G and 100 mg/ml streptomycin) at 37 °C in a humidified atmosphere with 5% CO_2_.

### Quantitative polymerase chain reaction

Total RNA was extracted from tissues and cells using TRIzol (Invitrogen, Carlsbad, CA, USA) according to the manufacturer’s protocol, and cDNA was synthesized using Primescript RT reagent (Takara, Shiga, Japan). qPCR was performed using a 7900 Real-Time PCR System (Applied Biosystems, Foster City, CA, USA) with Fast Start Universal SYBR Green Master (Takara). Relative BCL9 and VEGF-A expression were normalized to the level of *β*-actin expression. The primers used in this study were as follows: BCL9 forward: 5′-CCCCATCAAATGCTACAGCC-3′ and BCL9 reverse: 5′-TTTCAACCTGGCCCTTCAAAA-3′ VEGF-A forward: 5′-AGGGCAGAATCATCACGAAGT-3′ and VEGF-A reverse: 5′-AGGGTCTCGATTGGATGGCA-3′ *β*-actin forward: 5′-TGACGTGGACATCCGCAAAG-3′ and *β*-actin reverse: 5′-CTGGAAGGTGGACAGCGAGG-3′. All procedures were performed in triplicate.

### miRNA RT-PCR

Total RNA was extracted as above, and the cDNAs of miRNAs were reverse transcribed using the reverse translate kit PrimeScript RT Master Mix (DRR037A; Takara) according to the manufacturer’s protocol, with a specific miR-1301 primer. Sequence-specific primers for U6 and miR-1301 were synthesized by RiboBio (Guangzhou, China). Real-time PCR was carried out with SYBR Premix EX Taq II (Takara). The reactions were also performed using the 7900 Real-Time PCR System. The snRNA U6 was selected as an endogenous reference to calculate the relative expression levels of miR-1301 in each sample using the 2^−ΔΔka^ method. All experiments were performed independently in triplicate.

### Vector and lentivirus production and transfection

We modified the commercially available LV3-has-miR-1301-pre-microRNA vector, the lentiviral vector containing the BCL9 DNA sequence (pre-miR-1301 and LV-BCL9), LV3-has-miR-1301-sponge inhibitor vector and the lentiviral vector containing BCL9 siRNA hairpin sequence (miR-1301 inhibitor and BCL9-shRNA) constructs (Genepharma, Shanghai, China). An LV3 scrambled lentiviral construct (miR-NC) was used as a negative control. All vectors were verified by sequencing. The miR-1301-NC, pre-miR-1301, and miR-1301 inhibitor lentiviral vectors were used to infect cells at an appropriate multiplicity of infection when SMMC-7721 and Huh-7 cells had grown to 40%–50% confluence. Then, we added 5 *μ*g/ml polybrene (Genepharma) to the cells to increase the infection efficiency. Stable cell lines were selected using 7 *μ*g/ml puromycin (Sigma-Aldrich, St. Louis, MO, USA) for 1 week, when cells were analyzed for miR-1301 expression.

### Western blot

Total protein was isolated from cells after transfection, and protein concentration was measured using the BCA protein assay kit (Beyotime, Shanghai, China) followed by the manufacturer’s instruction. Samples were electrophoresed using 10% SDS-PAGE, then proteins were transferred to PVDF membranes (Bio-Rad, Hercules, CA, USA). The membranes were incubated with specific primary antibodies (1:1000) at 4 °C overnight after blocking in skim milk. Next, the membranes were incubated with HRP-conjugated anti-rabbit IgG antibodies (1:2000) at room temperature for 2 h. Immunoreactive bands were visualized using an enhanced chemiluminescence detection system. GAPDH was used as an internal reference. Western blots were quantified using Image Pro Plus version 6. Rabbit anti-BCL9, VEGF-A (Abcam, Cambridge, UK), *β*-catenin, *β*-actin and GAPDH (Cell Signaling Technology, Danvers, MA, USA) antibodies were used.

### ELISA for VEGF-A

The concentration of VEGF-A in supernatant was measured using the Quantikine human VEGF-A ELISA kit (Dakewei, Shenzhen, China), according to the manufacturer’s instructions. SMMC-7721 and Huh-7 cells transfected with miR-NC, pre-miR-1301 and miR-1301 inhibitor were seeded into six-well plates and cultured to 80% confluence, after which the cells were then switched to fresh medium. After 24 h, the cell culture supernatant was harvested and cell counts were performed after trypsinization. After collection, the medium was centrifuged at 2000 × *g* for 20 min at 4 °C to remove cellular debris. The concentration of VEGF-A in 100 *μ*l of supernatant was determined and normalized to the cell number. A serial dilution of recombinant human VEGF-A was included in each assay to create a standard curve.

### *In vitro* HUVEC tube -formation assay

Cells transfected with miR-NC, pre-miR-1301, and miR-1301 inhibitor were cultured as described above. When the cells reached 80% confluence, the culture medium was changed to serum-free DMEM. Following an additional 24-h culture, the supernatant was collected as conditioned medium and stored at −80 °C. For the tube-formation assay, each well of a 96-well plate was pre-coated with 50 *μ*l of Matrigel (BD Biosciences, Franklin Lakes, NJ, USA), which was allowed to polymerize for 30 min at 37 °C. HUVECs were suspended at a density of 2 × 10^5^ cells/ml in the different supernatants, and 100 *μ*l of the cell suspensions were added to each Matrigel-coated well. DMEM was used as the negative control. After 4 h, tube images were taken using a digital camera attached to an inverted phase-contrast microscope. The total tube length in each well was measured and calculated using Image Pro Plus.

### HUVEC migration and invasion assays

Cell migration and invasion assays were performed using a 6.5 mm chamber with 8 *μ*m pores (Corning, Corning, NY, USA). A cell suspension containing 2.5 × 10^4^ cells/ml was prepared in serum-free media, and 400 *μ*l of the cell suspension was added into the upper chamber. Subsequently, 600 *μ*l of the different conditioned media were added to the lower chambers. For invasion assays, the top chamber was coated with 100 *μ*l of 1 mg/ml Matrigel (BD Biosciences). After incubating for 36 h at 37 °C in a 5% CO_2_ humidified incubator, the cells that did not migrate through the pores and remained in the upper chamber were removed by scraping the membrane with a cotton swab. The migrated cells on the lower side of the membrane were stained with 0.1% crystal violet (Sigma-Aldrich) for 30 min at 37 °C, followed by washing with PBS and photographing 10 random fields of view at × 10 magnification. Cell numbers were counted and expressed as the average number of cells/field of view. Three independent experiments were performed.

### SMMC-7721 and Huh-7 migration and invasion assays

Cell migration and invasion assays were performed using a 6.5 mm chamber with 8 *μ*m pores (Corning). For migration assays, 3 × 10^4^ SMMC-7721-NC, SMMC-7721-pre-miR-1301, SMMC-7721-miR-1301 inhibitor, Huh-7-NC, Huh-7-pre-miR-1301, and Huh-7-miR-1301 inhibitor stable cells were suspended separately in serum-free DMEM and plated in the top chamber of the inserts. Then, 500 *μ*l of 10% serum-containing DMEM was added to the lower chamber of the well and the cells were allowed to migrate under chemotactic drive at 37 °C for 24 h; the cells in the upper chamber were then removed using cotton swabs. For invasion assays, 3 × 10^4^ cells were seeded on Matrigel-coated membrane inserts. Cells that successfully migrated to the underside of the membrane were stained with 0.1% crystal violet for 30 min at 37 °C, followed by washing with PBS, and counting using a light microscope at × 4 magnification in four randomly selected fields. The experiments were performed three times in triplicate.

### Wound healing assay

SMMC-7721 and Huh-7 cells (5 × 10^5^) were grown in six-well plates for 48 h until the cells were fully confluent. After non-adherent cells were washed away twice with PBS, a sterile 200- *μ*l pipet tip was used to make a uniform scratch in the center of the well. After 0 and 48 h, the distance between the wound sides was measured. Experiments were performed in triplicate.

### miRNA reporter luciferase assay

Cells were seeded into 24-well plates and co-transfected with 200 ng of pMIR-BCL9 or pMIR-BCL9-Mut and 100 ng of miR-1301 mimic or scramble miR mimic, and the pRL-TK plasmid (Promega, Madison, WI, USA) for internal normalization. Cells were harvested after 36 h and lysed using the lysis buffer (Promega). The luciferase reporter assay was conducted using the Dual-Luciferase Reporter Assay System (Promega), in accordance with the manufacturer’s instructions.

### Fluorescence *in situ* hybridization

MiR-1301 expression in HCC and adjacent normal tissues was detected by FISH. The mature human miR-1301 sequence is 3′-CUUCAGUGAGGGUCCGUCGACGUU-5′. We used LNA-based probes directed against the full length mature miRNA sequence. The 5′-FAM-labeled miR-1301 probe sequence was 5′-GAAGTCACTCCCAGGCAGCTGCAA-3′, and was purchased from BioSense (Guangzhou, China). The FISH assay was performed as previously described.^31^

### Tumor xenograft in animals

Four-week-old female BALB/c nude mice were purchased from the Department of Laboratory Animal Center of Nanjing Medical University. A total of 30 nude mice were randomly divided into six groups, and SMMC-7721-NC, SMMC-7721-pre-miR-1301, SMMC-7721-miR-1301 inhibitor, Huh-7-NC, Huh-7-pre-miR-1301, or Huh-7-miR-1301 inhibitor stable cells (2 × 10^6^ cells in 100 *μ*l PBS) were injected into the tail veins of the mice in the respective groups. After 6 weeks, the IVIS Imaging system (Caliper life Sciences, Hopkinton, MA, USA) was used to observe the occurrence of distant metastases. Care of experimental animals was in accordance with Nanjing Medical University Institutional Animal Care and Use Committee.

### Immunohistochemistry

All specimens were fixed in 4% formalin and embedded in paraffin. Sections were then cut and stained using previously described immunohistochemistry techniques.^32^ After blocking the endogenous peroxides and proteins, the 4-*μ*m sections were incubated overnight at 4 °C with diluted primary antibodies specific for BCL9, VEGF-A (Abcam) and CD31 (Cell Signaling Technology). Next, the slides were incubated with an HRP-polymer-conjugated secondary antibody at 37 °C for 1 h. The slides were then stained with a 3,3-diaminobenzidine solution for 3 min and counterstained with hematoxylin. Tumor slices were examined in a blinded manner. Three fields were selected to examine the percentage of positive tumors and staining intensities.

### Statistical analysis

Data are expressed as mean±standard deviation from at least three separate experiments. Statistical analyses were performed using SPSS v22.0 (SPSS Inc., Chicago, IL, USA). Qualitative data were analyzed by the chi-square test. Correlations were determined by Pearson correlation analysis. Independent *t*-tests were used to compare differences between two groups. One-way ANOVA with Bonferroni *post-hoc* tests were performed to compare differences among more than two groups. *P-*values <0.05 were considered statistically significant.

## Figures and Tables

**Figure 1:** miR-1301 was downregulated in HCC tissues and cell lines. (**a**) The levels of miR-1301 expression in 60-paired human HCC and adjacent normal tissues by qPCR. (**b**) The levels of miR-1301 expression in HCC cell lines and normal L02 cells. (**c**) The expression of miR-1301 in HCC specimens and adjacent normal tissues was detected by FISH assay (scale bars, 50 *μ*m). (**d** and **e**) SMMC-7721 and Huh-7 cells were transfected with specific pre-miR-1301 or miR-1301 inhibitor, respectively. Cells transfected with empty lentiviral vectors served as a negative control (NC). miR-1301 expression was analyzed by miRNA RT-PCR after transfection; cells transfected with empty lentiviral vectors were used as NC. *P<0.05, **P<0.01, ***P<0.001

**Figure 2:** miR-1301 negatively regulates HUVEC migration, invasion, and tube formation *in vitro*. (**a** and **d**) Tube-formation assays with HUVECs were performed with the indicated conditioned media. The network area was calculated using Image Pro Plus 6. (**b**, **c**, **e** and **f**) Transwell migration and Matrigel invasion assays with HUVECs were performed in each group. Cell migration and invasion capability were quantified as cell numbers. All experiments were performed three times, and data are presented as mean±S.D. values. *P<0.05 compared with controls

**Figure 3:** miR-1301 inhibits migration, invasion, and EMT in HCC cells. HCC SMMC-7721 and Huh-7 cells were transfected with LV3-has-miR-1301-pre-microRNA (pre-miR-1301) and LV3-has-miR-1301-sponge inhibitor (miR-1301 inhibitor) lentiviral constructs. An LV3 scrambled lentiviral construct (miR-NC) was used as a control. (**a**–**d**) Transwell assays were performed to determine cell migration and invasion and (**e**) wound healing assays corroborated these results. (**f**) Western blotting was used to examine the levels of EMT-related protein. Cell migration and invasion capability were quantified as cell numbers. All experiments were performed three times, and data are represented as mean±S.D. values. *P<0.05

**Figure 4:** miR-1301 inhibits VEGF expression. (**a**) qPCR was used to analyze the levels of VEGF-A expression in SMMC-7721 and Huh-7 cells transfected with miR-NC, the miR-1301 inhibitor, or pre-miR-1301. (**b**) VEGF-A protein levels were analyzed by western blotting. (**c**) ELISA was used to determine the VEGF-A concentration in the culture medium of SMMC-7721 and Huh-7 cells transfected with miR-NC, the miR-1301 inhibitor, or pre-miR-1301. *P<0.05

**Figure 5:** BCL9 was upregulated in HCC tissues and cell lines and is a direct miR-1301 target. (**a**) The levels of BCL9 expression were analyzed in 60-paired HCC and adjacent normal tissues by qPCR. (**b**) The levels of BCL9 expression in HCC cell lines and normal L02 cells. (**c**) BCL9 protein levels in HCC specimens and adjacent normal tissues as analyzed by immunohistochemistry. (**d**) The potential miR-1301 binding site in the BCL9 3′-UTR was computationally predicted by TargetScan. (**e**) The level of BCL9 expression in cells after transfecting pre-miR-1301 or miR-1301-inhibitor as detected by qPCR; cells transfected with empty lentiviral vectors were used as a negative control. (**f**) BCL9 and *β*-catenin protein levels in HCC cells transfected with miR-1301 inhibitor or miR-1301 overexpression lentivirus. (**g**) Dual-luciferase reporter assay analysis of the effects of miR-1301 expression on the activities of wild type and mutant BCL9 3′-UTR in 293 T cells. (**h**) A negative correlation between the levels of miR-1301 and BCL9 expression in HCC specimens (*P*<0.01). *P<0.05, **P<0.01, ***P<0.001

**Figure 6:** BCL9 overexpression eliminates the inhibitory effects of miR-1301 on HCC cell migration and invasion. (**a**–**d**) Western blotting was conducted to examine BCL9 protein expression in the indicated cells. (**e** and **f**) miR-1301 upregulation suppressed Huh-7 cell migration and invasion. The rescue experiments for miR-1301 overexpression were performed by ectopically expressing BCL9 (LV-NC). miR-1301 silencing was counteracted by downregulating BCL9, which was observed in SMMC-7721 cells. Cell migration and invasion capability were quantified as cell numbers. All experiments were performed three times, and representative data are displayed as mean±S.D. *P<0.05 compared with controls

**Figure 7:** miR-1301 overexpression suppressed HCC metastases *in vivo*. (**a** and **b**) Photographs of tumors were taken by the IVIS Imaging System (Caliper Life Science, Hopkinton, MA, USA). A representative luciferase signal was captured in each group 6 weeks after injecting SMMC-7721 and Huh-7 cells with negative control, miR-1301 overexpression and miR-1301 knockdown. (**c**–**e**) CD31, BCL9, and VEGF-A expression were analyzed in tumor tissues by immunohistochemistry; representative images are shown at × 20 magnification. Blood vessels were stained using anti-CD31 antibodies, and positively stained blood vessels were counted in five areas per slide to determine the maximum number of microvessels; 10 slides per experiment. The results are presented as mean±S.D. values. (**f** and **g**) The levels of miR-1301 expression in the metastatic tumors derived from nude mice were measured by qPCR. (**h**) The levels of BCL9 protein expression in the metastatic tumors derived from nude mice were measured by western blotting. *P<0.05

**Table 1:** Association between miR-1301 expression and clinicopathologic features of patients with hepatocellular carcinoma

		**miR-1301 levels**^a^		
**Variables**	**Number**	**Low (*n*=39)**	**High (*n*=21)**	***P-*value**
*Age (year)*				
<50	19	12	7	
≥50	41	27	14	0.839
				
*Gender*				
Female	25	15	10	
Male	35	24	11	0.493
				
*Tumor size (cm)*				
<5	38	26	12	
≥5	22	13	9	0.465
				
*Vascular invasion*				
No	33	17	16	
Yes	27	22	5	0.015*
				
*Edmondson grade*				
I+II	29	14	15	
III+IV	31	25	6	0.009*
				
*AFP*				
Negative	17	9	8	
Positive	43	30	13	0.218
				
*HBV infection*				
No	15	10	5	
Yes	45	29	16	0.876
				
*Cirrhosis*				
No	7	4	3	
Yes	53	35	18	0.643

Abbreviation: AFP, alpha-fetoprotein

*P<0.05 statistically significant difference

a The mean expression level of miR-1301 was used as the cutoff
